The article "Propofol Anesthesia Depth Monitoring Based on Self-Attention and Residual Structure Convolutional Neural Network" was published in 2022. Journal: Comput Math Methods Med.

# Propofol Anesthesia Depth Monitoring Based on Self-Attention and Residual Structure Convolutional Neural Network

**DOI:** 10.1155/2022/8501948

**Published:** 2022-01-29

**Authors:** Yachao Wang, Hui Zhang, Ying Fan, Peng Ying, Jun Li, Chenyao Xie, Tingting Zhao

**Affiliations:** ^1^Dept. Anesthesiol, First People's Hospital Xiaoshan, Hangzhou, Zhejiang, China; ^2^Department of Anesthesiology, Shulan (Hangzhou) Hospital Affiliated to Zhejiang Shuren University Shulan International, China

## Abstract

**Methods:**

We compare nine index values, select CNN+EEG, which has good correlation with BIS index, as an anesthesia state observation index to identify the parameters of the model, and establish a model based on self-attention and dual resistructure convolutional neural network. The data of 93 groups of patients were selected and randomly grouped into three parts: training set, validation set, and test set, and compared the best and worst results predicted by BIS.

**Result:**

The best result is that the model's accuracy of predicting BLS on the test set has an overall upward trend, eventually reaching more than 90%. The overall error shows a gradual decrease and eventually approaches zero. The worst result is that the model's accuracy of predicting BIS on the test set has an overall upward trend. The accuracy rate is relatively stable without major fluctuations, but the final accuracy rate is above 70%.

**Conclusion:**

The prediction of BIS indicators by the deep learning method CNN algorithm shows good results in statistics.

## 1. Introduction

In clinical anesthesia operations, as the depth of propofol anesthesia increases, explicit memory and implicit memory disappear one after another [1]. The patient still has implicit memory in the case of innocuous stimulus and unconsciousness. Different patients require different anesthesia operations. In the operation under epidural anesthesia (intraspinal anesthesia), in order to eliminate the nervousness of the patient, we avoid leaving unpleasant memories to the patient, and eliminate implicit memory [2]. For those who have poor general conditions and cannot tolerate deep intravenous general anesthesia (such as old age and shock). They should be anesthetized (composure) to at least 2 points on the OAA/S score to eliminate explicit memory [3].

The sedation stage during surgery is an important part of general anesthesia. Correct selection of the observation indicators for the sedation stage is an important step in anesthesia monitoring [4]. The static depth observation index includes BIS index, Narcotrend index, and entropy the index [5]. The entropy index can characterize the complexity of the signal and reflect the difference of signals in different states. The calculation process is relatively simple and has attracted more and more attention. The BIS monitor is currently the most authoritative anesthesia status monitor [6]. The BIS index is obtained by the BIS monitor and has a high degree of recognition in clinical anesthesia operations at home and abroad. However, its algorithm has high complexity and rich subparameters, which affects the reaction time of the indicator in a certain period of time. It is an indicator of the depth of sedation identified by the US FDA to monitor sedation. Studies show a good correlation of BIS with the concentration of multiple anesthetic drugs. However, the BIS is insensitive to the monitoring of the nociceptive stimuli and cannot respond immediately to the instantaneous changes in the EEG signals. Entropy index analysis of the complexity or “order” of the EEG was performed. As the anesthesia depth increases, the EEG data becomes more predictable or contains more “order,” with more order representing less complexity and a lower entropy index. However, when the depth of anesthesia was shallow, EEG data decreased order and irregularity increased. Unlike the BIS algorithm, the entropy index does not depend on the absolute frequency and amplitude range of the EEG, which is based on the analysis of the physiological condition of the measured patients. EMG signals need to be filtered from their data analysis in BIS monitoring, but entropy index monitoring is useful and in some cases more sensitive to the evaluation of awareness levels or analgesia than EEG. However, its algorithmic complexity is high and its subparameters are rich, which affects the reaction time of this index in a certain period of time. The BIS was used as a value indicating the depth of sedation. However, this value can change significantly in a short period of time due to interference from other instruments in the operating room (such as high-frequency electrical surgery), the effect of EMG on the patient frontal muscle and medication, and changes in the surgical position. Anesthesiologists often use this value to determine that it is true or false.

### 1.1. Reply to Solve

The field of anesthesia has significant advantages in the development and application of machine learning technology: various computer control systems, such as monitors, drug infusion systems, and anesthesia electronic medical record systems can be directly connected to each patient to collect a large amount of high-fidelity data in real time. Monitoring the depth of anesthesia has always been a key issue for anesthesiologists [7]. Insufficient depth of anesthesia leading to intraoperative awareness may have serious psychological effects on the patient, and overdose of anesthetic may prolong the recovery time of anesthesia and even cause irreversible damage to the patient [8]. Objective, noninvasive, and reliable monitoring of the depth of anesthesia is a challenge for clinical anesthesia.

Therefore, this paper proposes a new method of analyzing propofol anesthesia from two aspects of nine parameter indicators and BIS subparameters, based on self-attention and residual structure of the convolutional neural network.

First, we use Butterworth filter and other methods to preprocess the EEG signal and then use the manual feature extraction method mentioned in related theories to extract the sample entropy, sort entropy, frequency spectrum, and a ratio from the EEG signal. We analyze the characteristics of BIS parameters. BIS parameters are suitable for anesthesia monitoring, combined with a new method of convolutional neural network based on self-attention and residual structure to build a model, and combine different EEG signal parameters with machine learning algorithms to evaluate the anesthesia status can accurately quantify the patient's anesthesia status. This method does not need to refer to the age of the patient and the anesthetic drugs used and can reliably predict the depth of anesthesia. Compared with a single feature, this model can accurately estimate the depth of anesthesia with a higher prediction probability. The experimental results evaluated on the data set show that the method proposed in this paper provides better performance compared with ranking entropy, the ratio, and other traditional methods.

## 2. Related Work

### 2.1. Entropy Index

#### 2.1.1. Sample Entropy

The sample entropy (Sampan) was proposed by Richman and Moorman. The sample entropy can represent the complexity of a finite time series [9]. The larger the value of sample entropy, the more irregular the signal is reflected. Given a time series *x*(*i*), 1 ≤ *i* < N can reconstruct it into *N* − *m* + 1, a vector *x*_*m*_(*i*), which is defined as

(1) $$\begin{array}{c} x_{m}\left(i\right)=\left\{x\left(i\right),x\left(i+1\right),\cdots ,x\left(i+m-1\right)\right\},i=1,2,\cdots ,N-m. \end{array}$$

Let *d* be the distance between the vector *x*_*m*_(*i*) and *x*_*m*_(*j*) the formula as follows:

(2) $$\begin{array}{c} d_{ij}^{m}=d\left[x_{i}^{m},x_{j}^{m}\right]=\max\left(\left|x\left(\text{i}+k\right)-x\left(j-k\right)\right|\right),k=0,1,\cdots ,m-1. \end{array}$$

*C*_*i*_^*m*^(*r*) is the probability of *x*_*m*_(*j*) within the distance r of *x*_*m*_(*i*), which is calculated as

(3) $$\begin{array}{c} C_{i}^{m}\left(r\right)=\frac{n_{i}\left(m,r\right)}{N-m+1},i=1,N-m. \end{array}$$

Among them, *n*_*i*_(*m*, *r*) is the number of vectors *x*_*j*_ similar to *x*_*i*_, where *d*(*x*_*i*_, *x*_*j*_) ≤ *r*. When the embedding dimension is equal to *m*, the total number of template matches is

(4) $$\begin{array}{c} A\left(m,r\right)=\frac{\sum_{i=1}^{N-m}C_{i}^{m}\left(r\right)}{N-m}. \end{array}$$

Let *m* = *m* + 1, and repeat the above steps, the sample entropy of this time series can be expressed as

(5) $$\begin{array}{c} SampEn\left(r,m,N\right)=-\text{Ln}\frac{A\left(m+1,r\right)}{A\left(m,r\right)}. \end{array}$$

Ln is the natural logarithm. The sample entropy is affected by three parameters *r*, *m*, and *N*. *N* is the length of the time series, *r* is the threshold for determining the similarity of the pattern, and *m* is the length of the comparison sequence. In this paper, we set *N* = 500, *r* = 0.2, and *m* = 2, and the selection of parameters can be based on Bruhn's paper.

#### 2.1.2. Sort Entropy

Sorting entropy (PeEn) provides a simple and robust method for estimating the depth of anesthesia with low computational complexity. It quantifies the number of regularities in the EEG signal and takes into account the time sequence of these values. Given a time series *x*_*N*_ = [*x*_1_, *x*_2_, ⋯*x*_*N*_] with *N* points, *x*_*N*_ can be constructed as

(6) $$\begin{array}{c} x_{N}=\left\{x\left(i\right),x\left(i+\tau \right),\cdots ,x\left(i+\left(m-1\right)\tau \right)\right\},i=1,2,\cdots ,N-\left(m-1\right)\tau , \end{array}$$

where *τ* is the time delay and *m* represents the embedding dimension. Then, you can rearrange *x*_*i*_ in increasing order:

(7) $$\begin{array}{c} \left\{x\left(i+\left(j_{1}-1\right)\tau \leq x\left(i+\left(j_{2}-1\right)\tau \right)\leq \cdots \leq x\left(i+\left(j_{m}-1\right)\tau \right)\right.\right\}. \end{array}$$

The sequence of length *m* has *J* = *m*! permutations. Each vector *x*_*i*_ can be mapped to one of the permutations *J* = *m*! Next, the probability *p*_*j*_ of the *j*th permutation can be defined as

(8) $$\begin{array}{c} P_{j}=\frac{n_{j}}{\sum_{j=1}^{m!}n_{j}}. \end{array}$$

Among them, *n*_*j*_ is the number of occurrences of the *j*th arrangement. The sort entropy can be defined as

(9) $$\begin{array}{c} \text{PE}=\frac{\sum_{j=1}^{m!}P_{j}\log P_{j}}{\log\left(m!\right)}. \end{array}$$

The calculation of sort entropy depends on the length of the time series *N* and the time lag of *m*, where *N* = 500, *m* = 4, and *τ* = 1. The choice of parameters can be based on the paper by Su et al.

#### 2.1.3. Wavelet Entropy

Wavelet entropy is based on wavelet transform with multiple scales and directions. Choosing the appropriate wavelet base, the original signal will be generated according to different scales, where *C*_*j*_(*k*) is the decomposition coefficient of each scale *j* [10]. The wavelet energy *E*_*j*_ of the signal is defined as follows:

(10) $$\begin{array}{c} E_{j}=\overset{L_{j}}{\underset{k=1}{\sum }}{\left|C_{j}\left(k\right)\right|}^{2}, \end{array}$$

where *L*_*j*_ represents the number of coefficients under each decomposition scale. Therefore, the total energy of the signal can be expressed as

(11) $$\begin{array}{c} E_{t\text{otal}}=\underset{j}{\sum }E_{j}=\underset{j}{\sum }\overset{L_{j}}{\underset{k=1}{\sum }}{\left|C_{j}\left(k\right)\right|}^{2}. \end{array}$$

Then, we divide the wavelet energy by the total energy to get the relative wavelet energy at each scale *j*:

(12) $$\begin{array}{c} P_{j}=\frac{E_{j}}{E_{\text{total}}}=\frac{\sum_{k=1}^{L_{j}}{\left|C_{j}\left(k\right)\right|}^{2}}{\sum_{j}\sum_{k=1}^{L_{j}}{\left|C_{j}\left(k\right)\right|}^{2}}. \end{array}$$

Finally, the wavelet entropy can be calculated from the above:

(13) $$\begin{array}{c} S=-\underset{j}{\sum }P_{j}\log\left(P_{j}\right). \end{array}$$

#### 2.1.4. Band Ratio

The *α* ratio, *β* ratio, and (*β*-*α*) ratio is also used to monitor the depth of anesthesia. The *α* ratio is the logarithmic relative power of two different frequency bands, which can be calculated in the following way:

(14) $$\begin{array}{c} \alpha_{\text{ratio}}=\log\frac{E_{30-42.5\text{hz}}}{E_{6-12\text{hz}}}. \end{array}$$

The formula for *β* ratio and (*β*-*α*) ratio is as follows:

(15) $$\begin{array}{c} \beta_{\text{ratio}}=\log\frac{E_{30-42.5\text{hz}}}{E_{12-21\text{hz}}}.\\ {\left(\beta ‐\alpha \right)}_{\text{ratio}}=\log\frac{E_{6-12\text{hz}}}{E_{11-21\text{hz}}}. \end{array}$$

Among them, *α*_ratio_, *β*_ratio_, and (*β*‐*α*)_ratio_ represent *α* ratio, *β* ratio, and (*β*-*α*) ratio, respectively, and *E*_30−42.5hz_, *E*_6−12hz_, and *E*_11−21hz_, representing the spectral energy of the 30-42.5 Hz, 6-12 Hz, and 11-21 Hz frequency bands, respectively.

### 2.2. Time Collar Characteristics

Time-frequency analysis is a powerful tool that can decompose a signal into time and frequency components. Therefore, it provides a means for analyzing nonstationary signals (such as brain electrical signals). In the analysis of this kind of signal, people are often interested in the changes in frequency components over time, which is particularly important when analyzing sleep EEG [11]. In sleep EEG, many events (such as sudden waking) are measured by amplitude and the sudden change of frequency characteristics.

Short-time Fourier transform (STET) is the simplest form of time-frequency analysis. Usually, people only consider the squared amplitude of the STFT, and this squared amplitude is called a spectrogram. In order to calculate the short-time Fourier transform, the signal of interest is evenly divided into multiple short-term overlapping parts, and then, the data of each part is windowed and Fourier transformed. The result is a set of Fourier transforms at different points in time that reveals the changes in these spectral properties from one segment to another, which is the evolution of frequency over time. The time-frequency resolution of STFT is directly determined by the size of the window length: the smaller the window length, the higher the time resolution, and the lower the frequency resolution; the larger the window length, the lower the time resolution and the higher the frequency resolution. By increasing the size of the window length, the frequency resolution can be improved at the expense of reducing the time resolution [12]. It should also be noted that a longer window length may violate the quasistationarity assumption required by the Fourier transform.

Therefore, in addition to analyzing the stationarity of the previous signal, issues related to time and frequency resolution should also be considered. Due to its simplicity and ease of implementation, STFT has been widely used in sleep EEG analysis.

### 2.3. Common Feature Extraction Methods of EEG Signals

In some past studies of EEG signals, in terms of feature extraction methods, they can be divided into two different categories. The first is the method of extracting features based on manual design. This method requires prior knowledge of EEG analysis to extract the corresponding features. These methods first extract the most common features, such as the time domain, frequency domain, and time-frequency domain features of a single-channel EEG waveform. Then, we apply traditional machine learning algorithms, such as support vector machine (SVM), random forest, and neural network and train the model for the application you want to implement based on the extracted features [13]. The BIS monitor is currently the most authoritative anesthesia status monitor. The BIS index is obtained by the BIS monitor and has a high degree of recognition in clinical anesthesia operations at home and abroad. It integrates multiple EEG parameters into a single indicator, including *α* ratio, synchronization speed ratio (SFS), median frequency (MPF), and edge frequency (SEF). Narcotrend index compares and analyzes the data accumulated by itself and automatically classifies the extracted EEG signals to judge different states of anesthesia. However, the complexity of its algorithm is relatively high, which affects the reaction time of the indicator in a certain period of time.

Although these methods have achieved reasonable performance, they also have some limitations and require certain prior knowledge of sleep analysis. The second is a method based on automatic feature extraction (for example, deep learning algorithms), in which the machine automatically extracts relevant features (for example, CNN extracts time-invariant features from the original EEG signal).

### 2.4. Automatically Extracted EEG Signal Features

Most of the features are extracted manually, which requires a certain degree of expertise. In recent years, based on deep learning, the method of automatically learning features from EEG signals has become popular, and there are also many methods of automatic sleep stage classification based on deep learning [14].

Due to the powerful ability of deep learning to automatically learn features from data and the amazing progress of deep networks in many fields, people are interested in applying it to automatic sleep stage classification. Using various deep learning techniques to classify sleep stages, the results obtained have made significant progress. CNN is a classic algorithm of deep learning technology, and it is also often used for sleep stage classification tasks. The weight sharing mechanism of the convolutional layer makes the learned features have shift invariance, reduces the complexity of the model, and improves the generalization ability of the model. Therefore, it is usually used as a supplement to other network types, such as CNN and DNN. Independent CNN has also been used to learn the sequential features of sleep, usually in an end-to-end manner in the network [15].

### 2.5. Evaluation Indicators

Previously, that is, the sample entropy (SampEn), sorting entropy (PeEn), wavelet entropy, *α* ratio, *β* ratio, and (*β*-*α*) ratio, synch fast slow (SFS), median frequency (MPF), spectral edge frequency (SEF), BIS, and CNN+BIS, nine kinds of anesthesia state observation indicators are introduced and parameters are selected. In order to compare the relationship between these nine indicators and BIS, the correlation coefficient was calculated.

The correlation coefficient is a measure of the correlation between two time series *x*(*t*) and *y*(*t*). The formula is as follows:

(16) $$\begin{array}{c} \text{COR}\left(t\right)=\frac{\mathrm{cov}\left(x\left(t\right),y\left(t\right)\right)}{\sqrt{\mathrm{var}\left(x\left(t\right)\mathrm{var}y\left(t\right)\right)}}. \end{array}$$

In the formula, cov(*x*(*t*), *y*(*t*)) is the covariance of *x*(*t*) and *y*(*t*); var(*x*(*t*)) is the variance of *x*(*t*); and var(*y*(*t*)) is the variance of *y*(*t*).

The correlation coefficient describes the degree of correlation among the variables *x*(*t*) and *y*(*t*). The value range of COR (*t*) is [−1, 1]. If COR(*t*) > 0, then there is a positive correlation between *x*(*t*) and *y*(*t*). However, when COR(*t*) < 0, there is a negative correlation between *x*(*t*) and *y*(*t*). This study uses the absolute value of COR (*t*), namely ∣COR (*t*)∣ to measure the two indicators the degree of correlation between the two indicators. When the ∣COR (*t*)∣ value is greater than 0.8, it is highly correlated, 0.5 to 0.8 is moderately correlated, 0.3 to 0.5 is low correlated, and less than 0.3 indicates no correlation.

In addition, in order to compare the relationship between these 9 indicators and BIS indicators, we calculated the 9 indicator values of the EEG data of 20 patients and then calculated the correlation between them and the CNN+BIS indicators. The statistics of specific relevance are shown in Table 1.

According to the results in the table, the average correlation coefficients of ApEn, *α* ratio, SampEn, SFS, and CNN+EEG and BIS indicators are all higher than 0.6, indicating that these 6 indicators and BIS indicators have a high correlation during anesthesia. Among them, the correlation coefficient between CNN+EEG and BIS is the largest; indicating that among these nine indicators, CNN+EEG and BIS have the best correlation. Therefore, the parameters with better correlation with the BIS index are selected as the observation index of anesthesia state to carry out the parameter identification of the model.

## 3. Experiment

### 3.1. Research on Metabolic Model Based on Deep Learning

#### 3.1.1. Model Construction Ideas

Sheiner's PKPD model consists of two parts, namely, the PK model and PD model. However, the model parameters are greatly affected by individual differences, so there are still some differences between the theoretical model and the actual drug metabolism model. In response to these problems, this paper proposes a scheme of using deep learning algorithms to replace the traditional PKPD model. The concept of the model is shown in Figure 1.

Figure 1 is a conceptual diagram of the traditional PKPD model and the metabolic model based on deep learning. Among them, Figure 1(a) is a conceptual diagram of the traditional PKPD model. Among them, Ce represents the effect chamber concentration and Cp represents the blood drug concentration [16]. The covariates are the four physiological parameters of height, weight, gender, and age.  Figure 1(b) is a conceptual diagram of a metabolic model based on deep learning, where the input of the model is the feature index and covariate extracted from the EEG signal, and the output of the model is the depth of anesthesia index. In the end, the basis for judging the quality of the model training is the degree of fit between the index values output by the model and the actual index values.

#### 3.1.2. Introduction to CNN Algorithms

The concept of CNN was proposed by Yann at New York University in 1998. CNN is a deep learning algorithm, which has been widely used in image recognition and other fields. The structure of CNN mainly includes the input layer and hidden layer. The hidden layer is the focus of the CNN network. The hidden layer generally includes a pooling layer, a convolutional layer, and a fully connected layer. The convolutional layer and the pooling layer are unique to CNN [17].

Convolution operation is the focus of CNN. Under the action of the convolution kernel, the input data is subjected to convolution operation. Then, we add the deviation term to the obtained result, which can be input into the excitation function, and the value of the upper neuron can be obtained. The value at the (*i*, *j*) position on the upper layer is output by the *l*th convolution kernel on the *s* layer, which can be expressed as

(17) $$\begin{array}{c} x_{i,j}=f\left(w{\left(s\right)}_{j}∙I\left(i,j\right)+d\right), \end{array}$$

where *I*(*i*, *j*) is the feature of the convolutional layer, *f* is the activation function; *w*(*s*)_*j*_ is the *j*th convolution kernel on the s layer, and *d* is the deviation term.

#### 3.1.3. Optimize the Network

Convolution can optimize the complexity of the network through the following two parts in the calculation:

1. Sparse connection in the previous network, the layer connection of neurons is generally fully connected. However, on the CNN, sparse connections are used between layers. This is because in CNN, there is a strong correlation between the two neighboring layers, so the next layer only needs to be connected to the previous layer, that is, local connection. This will not lead to the occurrence of information loss, and can reduce the size of the CNN structural parameters. The sparse connection between two adjacent layers is shown in Figure 2

In Figure 2, the *m* layer is the hidden layer, and the *m* − 1 layer is the input layer. According to the above thoughts, it can be seen that the *m* − 1 layer only needs to be connected to the *m* layer.

(2) For weight sharing in CNN, filter parameters are shared [18]. That is to say, each convolution kernel performs convolution operation on the overall receptive field. The parameters of each convolution kernel have bias terms and weight coefficients. The weight sharing is shown in Figure 3

It can be seen from Figure 3 that the number of neurons in layer *m* is 3. In the figure, the weights of the lines connecting different positions are shared. You can use gradient descent to learn the shared weights without any changes. The advantage of weight sharing is that it has nothing to do with the location of feature extraction when extracting features. And the number of weight parameters of CNN can be reduced to a greater extent.

After the convolution operation, the maximum pool sampling method is used to reduce the size. By finding the largest feature parameter in this range, and then downsampling, new features are obtained. The features that have undergone downsampling still retain the effective information, and the reduction of the dimensionality is conducive to training. Setting the size of the pooling core to *m* × *m*, the method can be expressed as

(18) $$\begin{array}{c} f\left(x\right)=\max\left(x_{\left(i,i+m\right)\left(\text{j},j+m\right)}\right). \end{array}$$

Finally, the prediction result is output through the fully connected layer. The input of the fully connected layer is the feature output by the CNN, and the output is the value corresponding to the sample to be predicted. Then, the CNN output is

(19) $$\begin{array}{c} y_{r}=f\left(w∙y_{r-1}+b\right). \end{array}$$

#### 3.1.4. Autoencoder

Autoencoder (AE) can be understood as a system that tries to restore its original input; as shown in Figure 4, it is a type of neural network. The blue dashed box is the AE model, which consists of two parts, an encoder *f* and a decoder *g*. The encoder converts the input signal *x* into a hidden representation *Y*, and the decoder restores *y* to the output signal *x*′, which is the reconstructed *x*.

(20) $$\begin{array}{c} y=f\left(x\right),\\ x^{\prime }=g\left(y\right)=g\left(f\left(x\right)\right). \end{array}$$

The purpose of the autoencoder is to recover the input *x* as much as possible. In fact, the network usually focuses on the encoding of the intermediate layer or the mapping from input to encoding. In other words, when the forced code *y* is different from the input *x*, the system can also restore the original signal *x*; then, the code *Y* already carries all the information of the original data, which is an effective representation of the automatic learning of the original data.

#### 3.1.5. Self-Attention Mechanism

Data will be generated during the learning process. As the amount of data increases, it is particularly important to clean, analyze, and model these data. In the modeling process, accelerating the training of the model can save a lot of time and cost. Therefore, some scholars proposed the self-attention mechanism based on the attention mechanism of the human brain and successfully applied it in the field of natural language processing [19]. The idea of this model comes from the attention mechanism. The self-attention mechanism can realize parallel computing more easily than the attention mechanism. Its basic structure is shown in Figure 5.

First, we multiply the input text information by the corresponding weights to obtain *q*1, *k*1, and *v*1. The calculation process is as follows:

(21) $$\begin{array}{c} q\left(i\right)=W^{q}x\left(i\right),\\ k\left(i\right)=W^{k}x\left(i\right),\\ v\left(i\right)=W^{v}x\left(i\right), \end{array}$$

Among them, *W*^*q*^, *W*^*k*^, and *W*^*v*^ correspond to the weight matrices of *q*, *k*, and *v*, respectively; *i* = [0, *N*], and *N* is the size of the sample value. We perform the dot product operation on the obtained *qi* and *ki*, then normalize the result, and finally multiply the corresponding weight *v*(*i*) to get the output content, namely,

(22) $$\begin{array}{c} \alpha \left(1,i\right)=\frac{q\left(i\right)∙k\left(i\right)}{\sqrt{d}},\\ \tilde{\alpha }\left(1,i\right)=\exp\left(\alpha \left(1,i\right)\right)/\underset{j}{\sum }\exp\left(\alpha \left(1,j\right)\right),\\ b\left(i\right)=\underset{i}{\sum }\tilde{\alpha }\left(1,i\right)v\left(i\right). \end{array}$$

It can be seen from the calculation result of *b*(*i*) that the result value of each *b*(*i*) is related to the entire input sequence, which is also one reason why the self-attention mechanism can speed up the calculation in parallel. The above calculation process is expressed as a matrix:

(23) $$\begin{array}{c} \text{self}‐\text{Attention}\left(Q,K,V\right)=\text{softmax}\left(\frac{QK^{T}}{\sqrt{d_{k}}}\right)V. \end{array}$$

Among them, *Q*, *K*, and *V* are matrices formed by concatenating each of the above *q*(*i*), *k*(*i*), and *v*(*i*). Therefore, another reason for the acceleration of the calculation speed is that the essence of the attention mechanism is matrix calculation.

#### 3.1.6. Residual Network

With the continuous development of deep learning, the depth of the network is getting larger and larger. Although the accuracy of the model has been improved, a series of problems have arisen, such as gradient explosion and gradient disappearance. Initializing the weight parameters is particularly important. A reasonable weight value can prevent the parameters from entering the activation function saturation region, thereby reducing the problems of gradient disappearance and gradient explosion. However, the method of randomly initializing parameters is inefficient. He et al. [20] and others proposed a deep residual model (residual network (ResNet)), which not only solves the problem of gradient disappearance caused by deep networks but also solves the problem of network degradation. At the same time, the accuracy of the model has been improved. The basic residual structure is shown in Figure 6:

*x* is the information input, *H*(*x*) is the characteristic information output, *F*(*x*) is the residual, and its expression is

(24) $$\begin{array}{c} F\left(x\right)=H\left(x\right)-x. \end{array}$$

The information input *x* can be directly connected to the back access layer, so that the back access layer can learn the dual layer, so this connection is also called a shortcut connection. The residual structure increases the depth of the model through identity mapping. The basic operation is

(25) $$\begin{array}{c} x_{L}=x_{l}+\overset{L-1}{\underset{i=1}{\sum }}F\left(x_{i},w_{i}\right). \end{array}$$

*x*_*l*_ is the information representation of the features of the *L*th depth unit. When the residual value is 0, the residual network is equivalent to performing identity mapping, so as to ensure that the training accuracy of the model will not decrease. In fact, due to the complexity and diversity of the data, the residual value will not be 0, which is equivalent to the model is constantly stacking layers to better learn new features.

### 3.2. Parameter Setting of Each Layer

This paper uses the method of combining multiple convolutional layers, pooling layers, and superimposing the output of the fully connected layer to train the input data to be trained. In the setting of the training parameters of the CNN model, the learning rate is 0.01, and the ReLU function is used as the excitation function of each convolutional layer [21]. In the setting of the pooling layer, the maximum pool sampling method is used to reduce the output of the convolutional layer. We use SoftMax regression to output the predicted anesthesia state value.

In the model training, data from 93 groups of patients were used. First, it is divided into three parts: training set, validation set, and test set by random grouping. The grouping results are as follows: the training set includes 61 patient data (167772 data points in total), the validation set includes 16 patient data (68168 data points in total), and the test set includes 16 patient data (64793 data points in total), such as Figure 7. The specific data set characteristics are shown in Table 2.

In the part of the deep learning algorithm, a two-dimensional regressor is used. At this time, it is necessary to convert the one-dimensional EEG feature sequence into a two-dimensional matrix as the image format. Taking into account the *s* parameters as characteristic indicators and the four physiological parameters of height, weight, age, and gender, 48 indicator data were selected for combination in the same period, and they were sequentially combined into 576 numerical sequences. Then, we reshape 576 one-dimensional sequences into 24 × 24 two-dimensional matrices as the samples to be trained.

The sample set to be trained is used as the input of CNN, and the parameter settings and output of each layer are shown in Table 3:

### 3.3. Evaluation Indicators

In this paper, goodness of fit, mean square error, and average percentage error are used to evaluate the simulation prediction results. The calculation formula is as follows:

(26) $$\begin{array}{c} R^{2}=1-\frac{\text{SSE}}{\text{SST}}, \end{array}$$

(27) $$\begin{array}{c} \text{RMSE}=\sqrt{\frac{\sum_{i=1}^{n}\left(e_{i}-\bar{e}\right)}{n}}, \end{array}$$

(28) $$\begin{array}{c} \text{MAPE}=\overset{n}{\underset{i=1}{\sum }}\left|\frac{{\text{observed}}_{t}-{\text{predicted}}_{t}}{{\text{observed}}_{t}}\right|\times \frac{100}{n}. \end{array}$$

The meaning of these metrics is described as follows: The *R*^2^ coefficient in (26) is the goodness of fit of the model output, and the range is (0, 1). When the value of the goodness of fit is larger, it means that the result predicted by the model is closer to the true value; that is, the drug metabolism model obtained by training is more accurate [22–25]. Among them, SST is the sum of squared deviations, and SSE is the sum of squared residuals; RMSE in the Equation (27) is the mean square error of the training result. If its value is small, it means that the error of the training result is small. Among them, *e*_*i*_ is the test sample value, and $\bar{e}\;$is the average value of e; MAPE in the Equation (28) is the average percentage error.

## 4. Results

We use the CNN network to construct the drug metabolism model. We take the 8 characteristic parameters of SPE, ApEn, SampEn, SFS, *α* ratio, SEF95, MPF, SpEn, height, weight, age, gender, and BIS indicators extracted from the clinical EEG data of the patient as the input of the network model for training. Model training adopts a 5-fold cross-validation method, and the best and worst results of BIS prediction are shown in Figures 3–7 and Figures 3–8.

Figures 8 and 9, respectively, show the best and worst results of CNN model tracking BIS on the test set. Among them, the lighter solid line is the result of each iteration, the darker solid line is the result of smoothing the iteration result, and the black dashed line is the result of each verification. After every 30 iterations, the prediction results are verified once.

The curves in Figures 8 and 9, respectively, show the trend of the iterative verification accuracy of the CNN model on the test sample and the error trend with the number of iterations.

According to Figure 8, the whole process is displayed in 3 time periods, and each time period is iterated 57 times, a total of 171 iterations. The accuracy and error are verified every 30 iterations. It can be seen that as the number of iterations continues to increase; the accuracy of CNN in predicting BLS on the test set is generally on the rise, eventually reaching more than 90%. The overall error shows a gradual decrease and eventually approaches zero.

Figure 9 is also displayed in three time periods; each time period is iterated 75 times, a total of 225 iterations. The accuracy and error are verified every 30 iterations. It can be seen that as the number of iterations continues to increase, and the accuracy of the model for predicting BIS on the test set is generally on the rise. The accuracy rate is relatively stable without major fluctuations, but the final accuracy rate is above 70%.

Further, we analyzed the results of several representative data samples and drew the corresponding curves, as shown in Figure 10. It can be seen intuitively from Figure 10 that through the training of the CNN model, a better BIS curve prediction can be achieved.

It can be seen intuitively from Figure 10 that through the training of the CNN model, a better BIS curve prediction can be achieved.  Figure 10(a) is a BIS prediction tracing curve of a 39-year-old man, Figure 10(b) is a BIS prediction tracing curve of a 28-year-old woman, and Figure 10(c) is a BIS prediction of a 70-year-old man.  Figure 10(d) shows the BIS prediction tracking curve of a 65-year-old female. According to the comparative analysis of different ages, the fit of the drug metabolism model based on the CNN training model has a certain relationship with the age of the patient. The fit is better in the young and middle-aged, and the fit is poor in the old. From the comparative analysis of different periods of anesthesia, it can be seen that in the induction period of anesthesia, the fitting effect of the predicted results is poor, and there is a relatively large deviation from the actual BIS value. At the same time, when the data fluctuates greatly, the predicted effect of the model is not good. But as a whole, the prediction results are within the range available in statistics.

In order to make the predictable result of the model more accurate, the prediction results data of each stage of anesthesia were counted. This paper mainly uses *R*^2^ coefficient, RMSE, and MAPE to evaluate the prediction results. The statistical results are shown in Table 4.

It can be obtained from Table 4 that in the prediction results of the controlled object based on the CNN training model, the maximum goodness of fit value of the test data set is 93.34 (%), and the smallest is 66.72 (%). The maximum RMSE value is 6.89, the minimum is 4.04, the maximum MAPE value is 14.73 (%), and the minimum is 3.99 (%).When analyzing the different stages of anesthesia, it was found that the predictive model performed the most stable in the maintenance phase and slightly worse in the induction and recovery phases. But on the whole, the predictive effect is within the range available in statistics.

## 5. Discussion

The analytical ability of machine learning algorithms is extremely high, which is superior to classical statistics. In recent years, great breakthroughs have been made in the imaging diagnosis of pulmonary nodules [22], and while maintaining good sensitivity with higher specificity than traditional methods, [23] deep learning algorithms also have good prospects in the sedation monitoring of anesthesia. For the small- and medium-sized surgery of ASAI-II can obviously assist the anesthesiologist to make the appropriate judgment to reduce the work intensity; but for the patients with ASAIII-IV undergoing large surgery, the use of vasoactive drugs is more complicated due to the drastic hemodynamic changes, and how to improve the sensitivity and stability of the analysis under this conditions is the direction of our next study At the same time, it is necessary to pay attention to the shortcomings of artificial intelligence itself, such as the inability to empathize with the patient, the inability to understand the patient's acceptance of anesthesia and surgical methods, and the trust in intelligent medical care degree [24]. It is very difficult for anesthesiologists to understand the internal mechanisms of machine learning. Although the machine learning algorithm has been successful in various trials, it is difficult for clinicians to judge whether there will be errors inside the “black box,” so it may be difficult for the machine learning algorithm to gain the clinician's reliance. Finally, the necessary premise of machine learning algorithms is to collect a large amount of high-fidelity physiological monitoring data from patients [25]. If the data is incomplete, unstable, biased, or even wrong in the training process, it may produce wrong results and mislead the doctor to make wrong judgments.

Therefore, it is necessary to ensure that a large amount of high-quality data is available to promote the success of machine learning in terms of adaptive control [26]. At present, the most reasonable way to introduce artificial intelligence and machine learning into anesthesia practice is still to manage the use of a closed-loop control system of drugs during routine operations of patients to maintain a stable anesthetic drug maintenance [27]. However, artificial intelligence has entered the field of anesthesia as a stepping stone, which brings challenges to the future development of anesthesiologists, as well as opportunities for professional development. It can effectively reduce the workload of anesthesiologists and give doctors more time and energy to focus on the impact of the progress of the surgery on patients. Of course, AI cannot completely replace anesthesiologists; anesthesiologists have to be prepared for the change of work philosophy [28].

## 6. Conclusion

With the advent of the “big data” era, artificial intelligence technology and the information industry will play a huge role in promoting the development of human health. More and more machine learning technologies may enter perioperative medicine, affect clinical decision-making, and improve patient's prognosis. The intelligent machine algorithm's assessment of patients and precise control of anesthesia will provide patients with a more comfortable anesthesia experience. In-depth monitoring of anesthesia is of great significance to improving the quality of anesthesia and ensuring the safety and rehabilitation of patients during the surgical period. Systematically, we review the EEG signal analysis algorithm, first compare the advantages and disadvantages of these parameters in clinical application, then propose the ranking entropy index algorithm with excellent denoising ability, and introduce the reverse mapping neural network to correct and optimize the EEG double frequency index, anesthesia trend, and ranking entropy index, so order to more accurately realize anesthesia depth monitoring. This paper introduces deep anesthesia monitoring as a deep CNC learning algorithm. A combination of index parameters extracted from the EEG signals and BIS index data was used as input for training. The results show that its prediction of BIS indicators reflects better statistical results. This paper introduces a deep learning method CNN algorithm. The index parameter combination extracted from the EEG signal and the BIS index data is used as input for training. The results show that its prediction of BIS indicators reflects better results in statistics.

## Figures and Tables

**Figure 1:** Conceptual diagram of the model.

**Figure 2:** Sparse connection of two adjacent layers.

**Figure 3:** Schematic diagram of weight sharing.

**Figure 4:** Self-encoder structure.

**Figure 5:** Self-attention mechanism model.

**Figure 6:** Residual network structure.

**Figure 7:** Division of the data set.

**Figure 8:** The optimal result of CNN tracking BIS on the test set.

**Figure 9:** The worst result of CNN tracking BIS on the test set.

**Figure 10:** Predictive tracking curve of 4 patients.

**Table 1:** Correlation coefficients between different indicators and BIS indicators.

Index	SampEn	PeEn	WE	*α*_ratio_	*β*_ratio_
COR	0.608 ± 0.31	0.621 ± 0.28	0.394 ± 0.36	0.687 ± 0.20	0.596 ± 0.33
Index	(*β*‐*α*)_ratio_	SFS	MPF	SEF	CNN+EEG
COR	0.564 ± 0.22	0.607 ± 0.22	0.035 ± 0.44	0.342 ± 0.36	0.717 ± 0.14

**Table 2:** Data set characteristics.

	Training cohort	Validation cohort	Testing cohort
Quantity	61	16	16
Weight (kg)	68.8 ± 10.2 (54-87)	67.2 ± 9.5 (55-81)	74.4 ± 8.8 (59-93)
Gender (male/female)	46/17	11/4	11/4
Age	55.4 ± 12.1 (22-83)	49 ± 11.5 (36-72)	57.3 ± 10.4 (24-78)
Height (cm)	167.4 ± 5.2 (158-180)	166.5 ± 5.3 (162-178)	169.7 ± 4.6 (160-180)

**Table 3:** Parameter settings of each layer of CNN.

Layer	Layer type	Nuclear model	Stride	Number of zero-padded turns	Output feature map size	Number of output feature maps
1	Convolutional layer 1	3 × 3	1	1	24 × 24	16
2	Pooling layer 1	2 × 2	2	—	12 × 12	16
3	Convolutional layer 1	3 × 3	1	1	12 × 12	32
4	Pooling layer 1	2 × 2	2	—	6 × 6	32
5	Convolutional layer 1	3 × 3	1	1	6 × 6	64
6	Pooling layer 1	2 × 2	2	—	3 × 3	64
11	Output layer	—	—	—	—	1

**Table 4:** CNN's prediction result evaluation table.

Period of anesthesia	*R* ^2^ (%)	RMSE	MAPE (%)
Induction period	81.65 ± 9.5	7.1 ± 1.5	10.5 ± 3.0
Maintenance period	85.28 ± 8.8	5.2 ± 0.8	8.8 ± 2.5
Recovery period	80.33 ± 9.2	6.7 ± 1.2	9.8 ± 3.1
Whole paragraph	84.97 ± 8.4	5.5 ± 1.0	9.1 ± 2.8

## Data Availability

All data analyzed during this study are available from the corresponding author upon request.
